The article "Establishing and Validating an Aging-Related Prognostic Four-Gene Signature in Colon Adenocarcinoma" was retracted in 2024. Reasons: signs of a paper mill; suspected computer-generated content; unreliable results or conclusions; concerns about the data.

# Establishing and Validating an Aging-Related Prognostic Four-Gene Signature in Colon Adenocarcinoma

**DOI:** 10.1155/2021/4682589

**Published:** 2021-11-08

**Authors:** Lian Zheng, Yang Yang, Xiaorong Cui

**Affiliations:** ^1^Department of Gastroenterology, Third Affiliated Hospital (Jie'er Hospital), Chongqing Medical University, Chongqing, China; ^2^Department of Geriatrics and Secret Service, First Affiliated Hospital, Army Medical University, Chongqing, China

## Abstract

**Background:**

Aging is a process that biological changes accumulate with time and lead to increasing susceptibility to diseases like cancer. This study is aimed at establishing an aging-related prognostic signature in colon adenocarcinoma (COAD).

**Methods:**

The transcriptome data and clinical variables of COAD patients were downloaded from TCGA database. The genes in GOBP_AGING gene set was used for prognostic evaluation by the univariate and multivariate Cox regression analyses. The model was presented by a nomogram and assessed by the Kaplan-Meier curves and calibration curves. The drug response and gene mutation were also performed to implicate the clinical significance. The GO and KEGG analyses were employed to unravel the potential functional mechanism.

**Results:**

The Gene Set Enrichment Analysis result indicates that GOBP_AGING pathway is significantly enriched in COAD samples. Four aging-related genes are finally used to construct the aging-related prognostic signature: FOXM1, PTH1R, KL, and CGAS. The COAD patients with high risk score have much shorter overall survival in both train cohort and test cohort. The nomogram is then assembled to predict 1-year, 3-year, and 5-year survival. Patients with high risk score have elevated infiltrating B cell naïve and attenuated cisplatin sensitivity. The mutation landscape shows that the TTN, FAT4, ZFHX4, APC, and OBSCN gene mutation are different between high risk score patients and low risk score patients. The differentially expressed genes between patients with high score and low score are enriched in B cell receptor signaling pathway.

**Conclusion:**

We constructed an aging-related signature in COAD patients, which can predict oncological outcome and optimize therapeutic strategy.

## 1. Introduction

Colorectal adenocarcinoma is the third most commonly diagnosed malignancy and the second leading cause of cancer-specific death worldwide [1]. Colon adenocarcinoma (COAD) is the main subtype of colorectal adenocarcinoma and the dominative pathological subtype colon cancer, accounting for over 90% colon cancer [2]. Although increasing therapeutic advancements in the past decades, the survival of COAD patients is still far from satisfactory since the initial diagnosis is usually delayed [3]. Besides, COAD is characterized by rapid progression and metastasis, which may cause worse prognosis [4]. Recently, some studies have shown that the variation of gene expression occurs during colon carcinogenesis and progression. Nevertheless, precise genetic alteration accounting for the initiation and development of COAD is poorly understood [5]. Therefore, establishment of gene signatures can help to develop clinical therapeutic strategies to improve patient prognosis.

The article "Establishing and Validating an Aging-Related Prognostic Four-Gene Signature in Colon Adenocarcinoma" was retracted in 2024. Reasons: signs of a paper mill; suspected computer-generated content; unreliable results or conclusions; concerns about the data.

Aging is a process that biological changes accumulate with time and lead to increasing susceptibility to diseases like cancer. The incidence of colon cancer is elevated by age, which may result from cumulative impact of long-term carcinogen exposure and gene mutation [6]. The *in vivo* research reports that aged colonic mucosa is more sensitive to carcinogen by stimulating higher ornithine decarboxylase and tyrosine kinase activities [7]. However, on the other hand, the activation of some molecule like transcription factor Nrf2 can prevent increasing oxidative stress in aging but also promote colon cancer chemoresistance and radioresistance [8]. In this study, we first explore the association between aging gene set and COAD. Then, the aging-related prognostic signature is constructed by multivariate Cox regression. A prediction model is established to predict oncological outcome, chemosensitivity, and immune cell infiltration of COAD patients. A further functional evaluation under differential aging risk scores is performed to unravel underlying mechanism.

## 2. Materials and Methods

### 2.1. Data Procession

Transcriptome profiles and clinical metadata of COAD patients were retrieved from TCGA database (https://portal.gdc.cancer.gov/). Gene set “GOBP_AGING” was searched and downloaded from the Gene Set Enrichment Analysis- (GSEA-) MSigDB database (https://www.gsea-msigdb.org/gsea/msigdb). All the data was processed by R program version 4.0.0.

### 2.2. Exploration of the Aging Pathway

We sorted the transcriptional matrix and performed GSEA between normal tissues and tumor tissues by setting “GOBP_AGING” gene set as the enrichment pathway. Then, we extracted the expression of the aging-related genes in the pathway and separately performed differential expression analysis to find differentially expressed genes (DEGs) and univariate Cox regression to discover prognostic genes. Following this, we took an intersect of these two gene lists and got differentially expressed prognostic aging genes. The left aging genes were input to the String database to further explore their protein-protein interaction (PPI), and Pearson correlation test was performed to check the correlation of their expression and establish the correlation network.

The article "Establishing and Validating an Aging-Related Prognostic Four-Gene Signature in Colon Adenocarcinoma" was retracted in 2024. Reasons: signs of a paper mill; suspected computer-generated content; unreliable results or conclusions; concerns about the data.

### 2.3. Signature Construction

We firstly randomly split the COAD patients into training set and validation set at a ratio as 1 : 1. Then, we performed univariate Cox regression in training set to find the potential prognostic factors with *p* < 0.05 and carried out multivariate Cox regression to establish the prognostic signature in training group. Thus, each patient in both training set and validation set acquired a risk score according to the formula as follows: Riskscore = ∑_*i*=1_^*N*^(Exp(*i*)∙coef(*i*)); here, *i* represented the *i*th gene in the prognostic signature, Exp(*i*) represented the expression value of *i*, and coef(*i*) represented the coefficient of *i* in the signature.

### 2.4. Signature Verification and Immune Infiltration

Because the prognostic signature was constructed according to the data in training set, we set the medium value of risk score in training set as the cut-off to stratify patients in both training set and validation set. Then, log-rank survival analysis was performed, and the Kaplan-Meier-based survival curve was plotted to check the prognostic value of risk score. CIBERSORT algorithm was performed to emphasize the immune infiltration of each sample; then, we compared the infiltration between high-risk and low-risk patients to further investigate the differences in immunity.

### 2.5. Nomogram and Calibration Curves

Considering the effects of clinicopathological characteristics, we established a nomogram in the training group using age, gender, stage, and risk score. Then, this nomogram was examined in training set (internal cross-validation), validation set (external validation), and all patients (external validation). Notably, concordance index (C-index) was used to check the efficacy of this nomogram. The nomogram was assembled using R package “rms.”

### 2.6. DEGs, Mutation Atlas, and Drug Response between High- and Low-Risk Patients

DEGs between high- and low-risk patients were defined with the ∣logFC | >1 and false discovery rate (FDR) < 0.05. Then, GO and KEGG enrichment analyses were performed to investigate the significant functions of these DEGs, and the PPI network was used to investigate the interaction and screen hub genes. Besides, the mutation atlas between high- and low-risk patients was explored, and the drug response to cisplatin and cyclopamine with the formation in half maximal inhibitory concentration (IC50) was predicted by the R package “pRRophetic,” and finally, we compared the drug response between high- and low-risk patients to distinguish the potential beneficiaries to the chemotherapy [9].

The article "Establishing and Validating an Aging-Related Prognostic Four-Gene Signature in Colon Adenocarcinoma" was retracted in 2024. Reasons: signs of a paper mill; suspected computer-generated content; unreliable results or conclusions; concerns about the data.

### 2.7. Statistical Analysis

All the statistical analysis was processed by R program 4.0.0 and Statistical Product and Service Solutions version 24. In detail, the differential expression analysis was examined by R package “limma” [10]. The immune infiltration was emphasized by the R package “CIBERSORT” [11]. The difference between two survival curves was evaluated by log-rank test. The differences of infiltrating immune cells and drug sensitivity between high-risk and low-risk patients were assessed by Wilcoxon rank-sum test when a nonnormal distribution was shown; otherwise, the *t* test or separate variance estimation *t* test was applied according to the equality of variances. The *p* value less than 0.05 was considered significant difference.

## 3. Results

### 3.1. Identification of Aging-Related Prognostic Signature

A total of 453 COAD patients from TCGA database are included in the study. The year of initial pathological diagnosis ranged from 1998 to 2013. (Table 1 shows the basic characteristics of the patients: age, sex, stage, tumor stage, regional lymph node status, and distant metastasis. The patients are randomly divided into train cohort (*n* = 228) and test cohort (*n* = 225). We use the train cohort to identify the signature. First, the GSEA result indicates that GOBP_AGING pathway is significantly enriched in COAD samples compared with normal colon tissue (Figure 1(a)). The results indicate that the aging genes in the GOBP_AGING pathway participant in the initiation of colon adenocarcinoma. We explore the expression pattern of individual genes in GOBP_AGING pathway (Figure 1(b)). There are 33 significantly downregulated genes and 61 upregulated genes in tumor samples. Among the differentially expressed genes, 15 genes have prognostic value for overall survival of COAD patients with log-rank test *p* value less than 0.05 (Figure 1(c)). Nine genes are downregulated (TMP1, TWIST1, SERPINE1, ADA, CDKN2A, CGAS, AMH, FOXM1, and TERT), and six genes are upregulated (PPARGC1A, KL, PTH1R, ATP8A2, PAX5, and C1QA) (Figure 1(d)).

Univariate Cox analysis shows that 6 genes can predict overall survival in COAD patients: FOXM1, PTH1R, PAX5, KL, CGAS, and ATP8A2 (Figure 2(a)). We performed multivariate Cox regression analysis to identify the independent predictor. Then, the aging-related prognostic signature is constructed by four genes: FOXM1, PTH1R, KL, and CGAS (Table 2). Figures 2(b) and 2(d) show the distribution of risk score in train cohort and test cohort, respectively. COAD patients with high risk score have much lower overall survival rate than the patients with low risk score in both train cohort (*p* = 0.006) and test cohort (*p* = 0.013) (Figures 2(c) and 2(e)). Highly enriched aging genes may impair the survival of COAD patients.

The article "Establishing and Validating an Aging-Related Prognostic Four-Gene Signature in Colon Adenocarcinoma" was retracted in 2024. Reasons: signs of a paper mill; suspected computer-generated content; unreliable results or conclusions; concerns about the data.

A nomogram is then established using the signature, age, and stage to predict 1-year survival, 3-year survival, and 5-year survival of COAD patients (Figure 3(a)). The calibration curves for train cohort, test cohort, and all patients show that the nomogram can effectively forecast the actual survival probability (Figures 3(b)–3(d)). These results identify an aging-related prognostic signature consisted of 4 genes that can be used to perform prognostic prediction.

### 3.2. Clinical Implication for the Aging-Related Prognostic Signature

We apply the CIBERSORT algorithm to estimate 22 types of infiltrating immune cells. The significant estimation with *p* value less than 0.05 is used for further analysis. The infiltrating immune cell profile is illustrated in Figure 4(a). COAD patients with high aging-related risk have higher infiltration level of B cell naïve (*p* = 0.010), T cell CD8 (*p* = 0.010), and T cell regulatory (*p* = 0.045), but lower infiltration level of B cell memory (*p* = 0.017), macrophage M0 (*p* = 0.043), and mast cells activated (*p* = 0.027) (Figures 4(b)–4(g)).

Chemotherapy is the main treatment for COAD patients. We evaluate the relationship between the aging-related prognostic signature and drug sensitivity (Figures 5(a)–5(c)). Patients with lower risk score are more sensitive to cisplatin (*p* < 0.001) and cyclopamine (*p* = 0.011), rather than paclitaxel (*p* = 0.31). The result indicates that patients with low risk score may have longer survival receiving cisplatin or cyclopamine treatments.

We also evaluate the gene mutation status in high-risk patients and low-risk patients (Figures 5(d) and 5(e)). Patients with high risk score have much higher mutation rate of TTN (53% vs. 45%), FAT4 (26% vs. 21%), and ZFHX4 (24% vs. 19%), but lower mutation rate of APC (72% vs. 77%) and OBSCN (18% vs. 23%) than patients with low risk score.

### 3.3. Functional Variance between High-Risk Patients and Low-Risk Patients

We investigate the differential expressed genes between high-risk patients and low-risk patients to unravel their functional variance. A total of 191 genes are significantly different between two groups (Figure 6(a)). Only one gene is downregulated. The GO analysis shows the gene participant in B cell-related biological process, such as B cell activation, B cell receptor signaling pathway, and B cell-mediated immunity (Figure 6(b)). The KEGG result indicates that the genes are enriched in pathways like PI3K−Akt signaling pathway and B cell receptor signaling pathway. These findings reveal that B cell-related molecule and pathways are highly activated in high score patients.

The article "Establishing and Validating an Aging-Related Prognostic Four-Gene Signature in Colon Adenocarcinoma" was retracted in 2024. Reasons: signs of a paper mill; suspected computer-generated content; unreliable results or conclusions; concerns about the data.

The PPI network is employed to depict the interaction profile and identify the hub genes (Figure 7). The top 5 hub genes are CD19, SNAP25, CD22, MS4A1, and CD79B, which play a central role in colon cancer initiation and development.

## 4. Discussion

In this research, we establish an aging-related prognostic signature consisting of four aging genes: FOXM1, PTH1R, KL, and CGAS. Among the four genes, FOXM1 and CGAS are highly expressed in COAD samples, while KL and PTH1R are downregulated during COAD initiation. In COAD patients, the elevated four genes all predict shorter survival. The aging-related prognostic signature can distinguish COAD patients with different overall survival in both train cohort and test cohort. The signature can also recognize the patients who are more sensitive to cisplatin and cyclopamine. The patients with high risk score have higher infiltrating B cell naïve and activating B cell-related pathways such as B cell activation and B cell receptor signaling pathway.

FOXM1 is a proliferation-related molecular belonging to the FOX transcription factor family. It widely participates in pathological process of tumor development, proliferation, invasion, metastasis, and chemoresistance [12, 13]. FOXM1 is repressed during human aging to cause mitotic decrease and aneuploidy, which further leads to aging-related disease [14]. In colon cancer, studies show that overexpression of FOXM1 is observed in tumor samples and dysregulated activation of FOXM1 promotes cancer growth and progression [15]. The aberrantly elevated expression of FOXM1 is associated with poor survival of COAD patients [15, 16]. The cyclic GMP-AMP synthase (CGAS) is involved in aging by CGAS-STING signaling. During cell senescence, cytoplasmic DNA is accumulated through the CGAS-STING signaling to stimulate senescence-associated secretory phenotypes, which will cause downstream senescence responses [17, 18]. The CGAS can also sense cytoplasmic DNA escape from the nucleus due to DNA damage in cancer cells and prevent aberrant development of cells [19]. The deficiency of CGAS may lead to tumorigenesis. However, we found that the CGAS gene expression is much higher in COAD tumor samples compared to normal samples. The elevated CGAS expression is related to poor survival. The results may indicate that chronic inflammatory and aging accompanied by activating CGAS-STING signaling lead to the initiation of colon cancer. There may be a mechanism for cancer cell to escape the surveillance of CGAS-STING signaling.

Hypercalcemia is reported as a critical factor associated with the progress and metastasis of malignancies [20, 21]. In colon cancer, slightly activated intracellular Ca^2+^ signaling can promote the initiation and development of colon cancer. But persistent Ca^2+^ influx and Ca^2+^ overload can lead to tumor cell death [22]. PTH1R is type 1 receptor of parathyroid hormone, regulating the serum concentrations of calcium and phosphate. Our study reveals that PTH1R is slightly reduced in COAD samples compared to normal samples. However, in COAD patients, higher PTH1R level is associated with poor prognosis. Liu and colleagues also suggested that PTH1R was correlated to miRNA and DNA methylation during liver metastasis of colorectal cancer [23]. The Klotho (KL) gene is also a key regulator during the aging process. The mice with overexpression KL gene have longer survival [24]. It is also identified as tumor suppressor gene in colon cancer. Rubinstein and colleagues found that KL can stimulate the unfolded protein response to inhibit colon cancer proliferation and viability [25]. Therefore, the aging signature that is constructed in our research can effectively predict the prognosis of COAD patients and participant in the pathological process of COAD.

The article "Establishing and Validating an Aging-Related Prognostic Four-Gene Signature in Colon Adenocarcinoma" was retracted in 2024. Reasons: signs of a paper mill; suspected computer-generated content; unreliable results or conclusions; concerns about the data.

Aging genes also regulate chemosensitivity of COAD patients. Our study reveals that the aging-related prognostic signature is associated with cisplatin sensitivity. Recent research shows that FOXM1, the direct target of miR-320, can diminish chemotherapy sensitivity with higher expression [26]. In addition, we identified the relationship between aging and B cell-related pathways in colon cancer. The patients with high risk score have upregulated B cell-related pathways. We speculate that the aging genes regulate tumor proliferation, invasion, metastasis, and chemosensitivity through remodeling B cell immunity. Further research needs to identify the role of B cell in aging-related colon cancer.

## 5. Conclusions

In summary, we constructed an aging-related signature in COAD patients, which can predict oncological outcome and optimize therapeutic strategy.

## Figures and Tables

**Figure 1:** Evaluation of aging genes in colon cancer. (a) Gene Set Enrichment Analysis for colon cancer using GOBP_AGING gene set. (b) Volcano plot for aging genes in colon cancer. (c) Venn plot for differentially expressed aging genes and prognostic genes. (d) Heatmap for aging genes with prognostic value.

**Figure 2:** Identification of aging-related prognostic signature. (a) Univariate Cox analysis for significant aging genes. The distribution of risk scores and survival status of colon cancer patients with different risk scores in (b) train cohort and (d) test cohort. The survival curves for patients with high risk score and low risk score in (c) train cohort and (e) test cohort.

The article "Establishing and Validating an Aging-Related Prognostic Four-Gene Signature in Colon Adenocarcinoma" was retracted in 2024. Reasons: signs of a paper mill; suspected computer-generated content; unreliable results or conclusions; concerns about the data.

**Figure 3:** Establishment of an aging-related prognostic model to predict overall survival in colon cancer patients. (a) The nomogram presenting the aging-related prognostic model. The calibration curves in train cohort, test cohort, and all patients.

**Figure 4:** The differentially infiltrating immune cells in colon cancer patients with high risk score and low risk score. (a) Profile of infiltrating immune cells in colon cancer patients. Differentially infiltrating (a) B cell naïve, (c) B cell memory, (d) macrophage M0, (e) mast cells activated, (f) T cell CD8, and (g) T cell regulatory (Tregs) between high-risk patients and low-risk patients.

**Figure 5:** The sensitivity of high-risk patients and low-risk patients to (a) cisplatin, (b) cyclopamine, and (c) paclitaxel. Mutation frequency in (d) high-risk patients and (e) low-risk patients.

**Figure 6:** (a) Differentially expressed genes between high-risk patients and low-risk patients. (b) GO analysis and (c) KEGG analysis for differentially expressed genes.

**Figure 7:** The protein-protein interaction network for differentially expressed genes.

**Table 1:** Basic characteristics of COAD patients.

Covariates	Total (*n* = 453)	Train (*n* = 228)	Test (*n* = 225)
Age			
≤65	188 (41.5%)	86 (37.7%)	102 (45.3%)
>65	265 (58.5%)	142 (62.3%)	123 (54.7%)

Sex			
Female	214 (47.2%)	115 (50.4%)	99 (44.0%)
Male	239 (52.8%)	113 (49.6%)	126 (56.0%)

Stage			
Stages I and II	250 (55.2%)	133 (58.3%)	117 (52.0%)
Stages III and IV	192 (42.4%)	91 (39.9%)	101 (44.9%)
Unknown	11 (2.4%)	4 (1.8%)	7 (3.1%)

T			
T1-2	88 (19.4%)	53 (23.3%)	35 (15.6%)
T3-4	364 (80.3%)	174 (76.3%)	190 (84.4%)
Unknown	1 (0.2%)	1 (0.4%)	0 (0.0%)

M			
M0	332 (73.3%)	170 (74.6%)	162 (72.0%)
M1	64 (14.1%)	26 (11.4%)	38 (16.9%)
Unknown	57 (12.6%)	32 (14.0%)	25 (11.1%)

N			
N0	266 (58.7%)	139 (61.0%)	127 (56.4%)
N1-3	187 (41.3%)	89 (39.0%)	98 (43.6%)

**Table 2:** Components of aging-related prognostic signature.

Gene symbol	Coefficient	HR	95% CI	*p* value
FOXM1	0.010	1.010	1.003-1.018	0.007
PTH1R	1.445	4.243	1.321-13.630	0.015
PAX5	0.333	1.396	0.980-1.987	0.064
KL	0.174	1.190	1.029-1.377	0.019
CGAS	0.181	1.198	1.051-1.366	0.007
ATP8A2	-2.94	0.053	0.001-2.745	0.145

## Data Availability

All original data that supports the findings of the research can be available from the corresponding author upon reasonable request.
